RETRACTED

# A model study of teaching method reform of computer laboratory course integrating internet of things technology

**DOI:** 10.1371/journal.pone.0298534

**Published:** 2024-04-18

**Authors:** Xiao Zhou, Ledan Qian, Haider Aziz, Marvin White

**Affiliations:** 1 Information Technology Center, Wenzhou University, Wenzhou, Zhejiang, China; 2 College of Mathematics and Physics, Wenzhou University, Wenzhou, Zhejiang, China; 3 College of Administration and Economics, Tikrit University, Tikrit, Salahdin, Iraq; 4 Department of Information Engineering, Southern University and A&M College, Baton Rouge, Louisiana, United States of America; TU Wien: Technische Universitat Wien, AUSTRIA

## Abstract

The Internet of Things (IoT) is gradually changing the way teaching and learning take place in on-campus programs. In particular, face capture services improve student concentration to create an efficient classroom atmosphere by using face recognition algorithms that support end devices. However, reducing response latency and executing face analysis services effectively in real-time is still challenging. For this reason, this paper proposed a pedagogical model of face recognition for IoT devices based on edge computing (TFREC). Specifically, this research first proposed an IoT service-based face capture algorithm to optimize the accuracy of face recognition. In addition, the service deployment method based on edge computing is proposed in this paper to obtain the best deployment strategy and reduce the latency of the algorithm. Finally, the comparative experimental results demonstrate that TFREC has 98.3% accuracy in face recognition and 72 milliseconds in terms of service response time. This research is significant for advancing the optimization of teaching methods in school-based courses, meanwhile, providing beneficial insights for the application of face recognition and edge computing in the field of education.

## 1. Introduction

The Internet of Things (IoT) is a network that combines sensing technology that can sense the world, radio frequency technology that can send signals, network connection technology for thing-to-thing communication, and embedded system technology for controlling devices, aiming to realize the interconnection of things with things and things with people [1]. In the field of education, the wide application of IoT technology has brought about a sea change in teaching and learning. By connecting various devices, sensors and networks, IoT offers many new possibilities for education [2]. Teachers are utilizing IoT technology to better understand their progress and level of understanding of their students. For example, through face-capture services, instructors identify the concentration level of their students with timely adjustments to teaching strategies in response and provide personalized instruction. In addition, through connected devices and networks, students access learning resources, participate in online discussions, and collaborate remotely with teachers whenever appropriate [3].

RETRACTED

In light of this, terminal cameras were installed into each seat monitor in the computer lab class [4]. Using a face recognition algorithm, features such as the direction of the student’s gaze, facial expression and head posture were automatically captured and analyzed. In this way, the student’s level of concentration is determined. If there are behaviors such as taking the face off the screen, looking down, shading, or closing the eyes for a long time, the algorithm automatically issues a warning to alert the teacher that the student needs to be given extra help. This technology helps the instructor to better understand the student’s learning status, identify problems, provide assistance in a timely manner, and improve teaching effectiveness [5].

However, face capture is a data-intensive service that requires a substantial amount of resources to process face image data, which leads to latency in IoT services [6]. The traditional cloud computing model transmits the data to be processed within a remote server, which increases the network transmission time and computational latency [7–9]. To solve this problem, edge computing is introduced to face capture services. The edge servers are directly connected to the camera devices, and face analysis algorithms are executed locally. Ultimately, edge computing reduces the network latency and decreases the response time of the face recognition service [10]. Furthermore, in educational environments where IoT technologies are employed, appropriate cybersecurity measures have to be put in place to protect the data of students from unauthorized access and attacks. Therefore, edge computing technologies process the data locally, reducing reliance on cloud servers to improve data security and privacy protection.

There has been relatively limited research on edge computing-based face recognition services for IoT environments [11]. Moreover, since face capture services have a wide range of applications in recognizing the concentration level of students, developing a face recognition service for IoT environments has become necessary research [12]. In addition, most currently available face recognition models based on edge computing concentrate on consumer scenarios such as smart homes, which still need to meet the actual demand for face capture services in education [13].

RETRACTED

Therefore, in this paper, an edge computing-based pedagogical model of face recognition for IoT devices called TFREC is proposed to solve the problem of face recognition service in the IoT environment. First, a three-layer cascaded convolutional neural network is used to model the face recognition problem to achieve dynamic recognition of facial features at IoT terminals. Then, to cope with the challenge of response latency, this paper incorporates edge computing and dynamic service deployment strategies. Finally, extensive simulation training is conducted to evaluate the performance of TFREC in terms of face recognition accuracy and service delay. The main contributions of this paper are as follows.

1. Proposed the TFREC model, which uses a three-layer cascaded convolutional neural network to achieve face recognition for IoT terminals, effectively recognizing facial features.
2. Utilized edge computing technology, the face recognition task is placed on edge servers closer to the user’s device, reducing data transmission and processing latency for improved response time.
3. Combined with dynamic service deployment strategy, face recognition service is dynamically deployed according to network state and device load to optimize response time and resource utilization. This strategy ensures that the resource allocation is adjusted despite high device loads, thereby efficiently providing face recognition services.
4. Evaluate TFREC through a large number of simulation experiments to verify that it has 98.3% accuracy in face recognition, the ability to meet large-scale task requirements in terms of service latency.

The paper structure is as follows. Section 2 discusses related work. Then, a specific algorithmic model is presented in Section 3. Section 4 presents a comparative analysis of simulation experiments and evaluations. The paper is concluded in Section 5. Finally, the limitations of the approach and future work to be carried out are discussed in Section 6.

## 2. Related work

### A. Methods of teaching courses in IoT

Using standardized methods is an important tool in order to ensure the quality of teaching and to optimize the teaching process. However, the large amount of data generated during the teaching process (e.g., attendance, classroom performance, assignments, and test results) usually have to be handled manually, with a certain degree of randomness, and is difficult to accurately reflect a situation in which a teacher is working. To cope with these problems, researchers have proposed a series of teaching management systems and methods based on IoT technology.

In particular, Wang et al. [14] proposed a university teaching management system based on integrated biometrics and IoT technology, which reduces the workload of teachers in the teaching process and improves the credibility and controllability of the data through the collaboration of data collection devices and the whole system. Upon this basis, Zhang et al. [15] constructed a teaching performance management system based on AIoT, which captured multimodal classroom behavioral data of teacher and student behaviors in real time to monitor the classroom teaching process. In terms of experimental teaching, Lei et al. [16] integrated the flipped classroom into the teaching of IoT development and applied it to the whole semester. Moreover, to guarantee the transmission security of teaching resources in the process of experimental teaching, He et al. [17] proposed a flipped classroom teaching method based on IoT technology for edible mushroom cultivation experiments and designed a secure convergence algorithm to improve the transmission efficiency of teaching resources.

RETRACTED

### B. Service deployment strategies under edge computing

In IoT environments, when edge servers need to serve a large number of users at the same time, the edge servers suffer from a serious interference problem, which reduces the service data transfer rate and leads to service blocking. In this regard, Qi et al. [18] proposed a model-free distributed deep reinforcement learning deployment algorithm for solving multi-objective optimization problems. The algorithm coordinates edge resources and achieves optimal service deployment through deep reinforcement learning. On this basis, Chen et al. [19] investigated the service deployment and application allocation problem in regional edge computing IoT, proposing a cooperative service deployment and application allocation algorithm to determine the final edge service deployment strategy. For the response latency problem, Li et al. [20] investigated a genetic algorithm-based microservice placement method, which effectively achieves low latency and load balancing by placing microservices on edge servers in a reasonable manner, thus reducing the transmission latency between microservices and server load. In addition, Zhao et al. [21] efficiently solves the application deployment problem and improves the quality of service by adopting a deployment prioritization greedy algorithm with a divide-and-conquer strategy.

### C. IoT face recognition in a cloud environment

Face detection is one of the most important operations in the field of digital image processing, which is used in many industries to solve security problems and save manual search time. Sumathi et al. [22] proposed a unique face recognition paradigm that utilizes the IoT security environment to identify specific criminal behaviors. Sistu et al. [23] proposed a framework for smartphone activation of secure access to closed indoor environments. Furthermore, to address the problem of massive data, Amin et al. [24] proposed an integrated framework utilizing IoT and cloud computing to develop a distributed face recognition scheme to support decentralized surveillance systems. On this basis, Abdulaziz et al. [25] utilized a time-stacked convolutional denoising self-encoder and an optimized Siamese convolutional gradient network to extract local features of face pose and expression changes and perform face recognition.

RETRACTED

However, as shown in Table 1, relatively scarce research has been conducted in the area of edge server deployment for face recognition services in IoT, while the application of joint learning in this area has not yet been widely adopted. Therefore, to address the problem of face recognition service deployment in teaching environments, this paper takes the IoT environment as a framework and deploys face capture service using a convolutional neural network, thereby improving the accuracy of recognition. Meanwhile, in order to adapt the real-time principle in the real teaching environment, the optimal edge server deployment strategy is proposed to reduce the service time delay.

**Table 1:** Main contributions in the literature.

Literature	Methodologies	Main Contributions	Performances	Data Set
Qi et al. [18]	A model-free distributed deep reinforcement learning deployment algorithm	Optimizing service deployment	Ensures balanced utilization while being able to reduce user latency	With 5 edge nodes and 10 microservice functions
Chen et al. [19]	A cooperative service deployment and application allocation algorithm	Optimizing service deployment	Most tasks are assigned to locally deployed elastic cloud servers, freeing up forwarding load on network switches	10 RANs and 800 IoT nodes
Li et al. [20]	A genetic algorithm-based microservice placement method	Optimize response latency	Latency and load balancing	13 edge servers for 15 microservice tasks
Zhao et al. [21]	A deployment prioritization greedy algorithm	Optimizing service deployment	Efficiently solve application deployment problems and improve quality of service.	Location information for 1464 real base stations and 174305 anonymous users
Sumathi et al. [22]	A unique face recognition paradigm	Optimize response latency	Face Recognition Methods Achieve 98.5% Accuracy Rate	1000 face images
Sistu et al. [23]	A framework for smartphone activation of secure	Constructing an IoT environment	91.75% accuracy in testing masks	511 images of faces wearing masks
Amin et al. [24]	An integrated framework utilizing IoT and cloud computing	Optimize decentralized monitoring	Detects and matches specific face images from a series of images captured by a video surveillance camera.	cloud data
Abdulaziz et al. [25]	A time-stacked convolutional denoising self-encoder and an optimized Siamese convolutional gradient network	Optimize Face Recognition	Minimized face recognition time with 99.75% accuracy rate	ORL data sets

RETRACTED

## 3. Method for IoT face recognition model based on edge environment

### 3.1 Definition of the problem

Face capture service is admittedly a data-intensive task that requires substantial resources to process face image data, leading to delays in IoT services. In addition, there is noise in the original face image in terminal monitoring, which can affect the detection accuracy of the face model, thus resulting in facial features not being effectively recognized.

### 3.2 Overall system construction

The main objective of this paper is to utilize a three-layer cascaded convolutional neural network deployed in an IoT edge server to efficiently process face image data from end devices and achieve real-time detection of features such as the direction of the student’s gaze, facial expression, and head posture [26]. By establishing a distributed face recognition system, the teacher more accurately understands the learning status of the students with timely detection of possible problems, thereby providing appropriate assistance to improve the teaching effect. By dynamically deploying the model in front of the terminal, the real-time response of the system is realized, moreover, the dependence on the central server is reduced, improving the performance and reliability of the system [27]. The specific system construction is shown in Fig 1.

**Fig 1:** Architecture of a distributed face recognition system for laboratory.

As shown in Fig 2, the traditional one-by-one matching method is time-consuming when facing amounts of massive face data [28]. Therefore, this paper adopted the computational method of distributed task allocation to shorten the time of matching the feature information of the face to be queried with the feature information in the face library [29]. In order to achieve this goal, this paper designs the following three steps: a) Face recognition and data acquisition: The face data to be queried is obtained by recognizing and acquiring faces in the terminal data. b) Fast face feature extraction: The face data to be queried is subjected to fast face feature value extraction to obtain its unique feature description information. c) Distributed Matching and Verification: The face features to be queried are matched and verified with the data in the face library to realize efficient distributed computing. By organically combining these three steps, the framework in this paper is able to significantly decrease the matching time and improve the efficiency during face recognition testing [30].

RETRACTED

**Fig 2:** Application of face recognition methods based on distributed technology to processes.

As shown in Fig 3, after the server calculates the feature values of the face photos transmitted from the terminal equipment, it quickly sends MapReduce jobs to the cluster in Fig 3, where the cluster splits the face library together with the recognized feature values in which the Map stage is responsible for splitting the face and recognizing the feature values while calculating the similarity, then through the Reduce process, the similarity is summed up and sorted, exporting the maximum similarity.

**Fig 3:** Distributed recognition matching flowchart.

To facilitate the understanding of the model formulas, the main symbols in the TFREC model algorithm are explained as shown in Table 2.

**Table 2:** Description of the main symbols in the formulas.

Symbols	Clarification	Symbols	Clarification
$T_{k,i}^{0}$	Upload Latency	$y_{i}^{\text{det}}$	The label for the image
$T_{k,i}^{1}$	Propagation Latency	$p_{i}$	Face recognition probability
$T_{k,i}^{2}$	Download Latency	${\hat{y}}_{i}^{box}$	Algorithm to detect image borders
$D_{k,i}$	The amount of data uploaded	${\hat{y}}_{i}^{mark}$	Algorithm detects image coordinate points
$D_{k,i}^{\prime }$	The amount of data downloaded	$y_{i}^{box}$	Actual image border
$\tilde{\lambda }$	Propagation rate	$y_{i}^{mark}$	Actual Image Coordinate Points
λ	Transfer rate	$b_{i}$	Face Candidate Box

### 3.3 Modeling dynamic deployment in edge computing

Network latency is an important metric for evaluating service performance in edge computing, which directly reflects the response time of service requests. In the experimental course teaching, the delay of model data during transmission is reduced in order to optimize the deployment resources of the service. Thereby, the latency of multiple students *S*_*k*_ to initiate a request to the face recognition service *A*_*i*_ is calculated by the following formula:

$$T_{k,i}=T_{k,i}^{0}+T_{k,i}^{1}+T_{k,i}^{2}$$ (1)

where $T_{k,i}^{0}$ and $T_{k,i}^{2}$ denote the delay time for the terminal device to upload the acquired Sk image data and download the final result, respectively, $D_{k,i}$ and $D_{k,i}^{\prime }$ denote the amount of data uploaded and downloaded by *A*_*i*_, respectively, and *λ* is the data transfer rate.

$$T_{k,i}^{0}=\frac{D_{k,i}}{\lambda },T_{k,i}^{2}=\frac{D_{k,i}^{\prime }}{\lambda }$$ (2)

$T_{k,i}^{1}$ is the propagation delay, which is caused by different services being placed on different edge servers and the services communicating with each other, as shown in Eq (3):

$$T_{k,i}^{1}=\frac{1}{\tilde{\lambda }}\times \sum_{l=1}^{\left|A_{i}\right|-1}(E_{l},E_{l+1})$$ (3)

where $\tilde{\lambda }$ denotes the propagation rate, except in the teaching environment where the different edge servers are configured in almost the same location, thus the propagation delay is 0.

RETRACTED

In addition, the real-time face request service has a high request frequency nature and requires redundant deployment in edge servers. Therefore, a discrete algorithm is used to calculate the distributed extensiveness SD, with lower values indicating more intensive services, as shown in Eq (4):

$$SD=\sqrt{\frac{\sum_{i=1}^{n}{\left[(x_{i}-\bar{x})+(y_{i}-\bar{y})\right]}^{2}}{n-1}}$$ (4)

To further measure the degree of service aggregation and to determine the number of redundant instances, this chapter uses an affinity propagation algorithm (AP) to perform clustering analysis, where a higher number of clustered results after clustering indicates a relatively wider distribution. Thereby, according to Algorithm 1, the service priority of each end device is calculated and ranked.

**Algorithm 1:** Service Prioritization

**Input:** student set *U*, application set *A*, service set *S*

**Output:** prioritized set of services S

 **Initialize Rank** *R* = (*R*_1_, *R*_2_, *R*_3_,…, *R*_S_)

 **For** *each j* **in** *S* **do:**

  Calculate the distribution *R*_*j*_ of requests for service *S*_*j*_ based on *U*, *A*

  *C*_*j*_ = *SD*(preference = *r*_*j*_.*request*)

  *S*_*j*_ = *sum*(*r*_*j*_.*request*)

  *R*_*j*_ = *C*_*j*_ + *S*_*j*_

 **End**

 Reorder *S* from largest to smallest based on *R*

 **Return** *S*, Deploy face recognition from **Algorithm 2** to *S*

Algorithm 1 calculates the priority of a service based on the distribution of demand for the service and the priority of the service in each end device. Its time complexity is divided into two parts, the first is to calculate the demand distribution of the service for each terminal device and the demand of the service in each application. Assuming that the number of terminal devices is U and the number of applications is A, the time complexity of this step is O(UA). The next step is to calculate the priority of the service, and the total priority of each service is calculated based on the distribution of the demand for the service by end devices and applications and the priority of the service itself. Assuming the number of services is S, the time complexity of this step is O(S). Therefore, the total time complexity of Algorithm 1 is O(UA + S).

RETRACTED

After prioritizing the services, dynamic deployment of the redundant number of instances of each service is required, depending on the situation. Specifically, in case no face image is captured by the current device, none of the service resources are allocated to the device. If multiple faces are detected by the end device, then the system will dynamically divide the computing resources of more edge servers to meet the demand of the face recognition algorithm. Ensure the optimal utilization of resources to provide proper service support for individual devices.

Therefore, the default redundancy value of the daily edge server is set to *N*. The $b_{j}^{0}$ represents the spare computing resources when assigning service *S*_*j*_, and the $b_{j}^{1}$ expresses the current running computing resources when assigning service *S*_*j*_, which is expressed as shown in Eqs (5–7) [31]:

$$b_{j}^{0}=b-\sum_{t=1}^{j-1}\left(c_{t}\times n_{t}\right)-\sum_{t=j}^{\left|S\right|}\left(c_{t}\times N\right)$$ (5)

$$b_{j}^{1}=c_{j}\times (N+c_{j}^{R})+b_{j}^{0}\times f_{j}$$ (6)

$$n_{j}=b_{j}^{1}/c_{j}$$ (7)

Where *n*_*j*_ is the number of redundant instances of the dynamically allocated service *S*_*j*_, *c*_*j*_ stands for the number of cluster result centers, and *f*_*j*_ denotes the ratio of the currently deployed computational resources of the service to the total service computational resources, which is computed as shown in Eq (8):

$$f_{j}=\left\{\begin{array}{ll} \frac{c_{j}}{\sum_{t=1}^{\left|S\right|}c_{t}}, & if\;b_{j}^{0}\geq 0\\ 0, & 0 \end{array}\right.$$ (8)

Eventually, service requests are dynamically deployed under the total resources *b*, to achieve real-time allocation of redundant instances *n*_*j*_ for the service *S*_*j*_ according to different environmental conditions.

### 3.4 Face recognition algorithm based on MTCNN

As shown in Fig 4, MTCNN is composed of three layers of cascaded convolution. First is the P-Net, which performs a fast face region filtering on the whole image by means of a shallow CNN network. Second is the R-Net, which is a layer trained to accurately localize the positions of facial feature points of the face and to filter and fine-tune the candidate frames using a deeper layer of convolutional neural network. In addition is O-Net, to further screen and refine the face candidate frames by combining the first two layers of network detection. Eventually, the output includes face regions, keypoints, pose estimation, etc. by continuously performing screening and adjustment. The cascade structure of MTCNN can effectively improve the accuracy of face detection and keypoint localization.

RETRACTED

**Fig 4:** Flowchart of MTCNN three-layer cascade.

The MTCNN face detection algorithm filters the face candidate frames by applying the Non-Maximal Suppression (NMS) algorithm. The algorithm decides whether or not to retain the detection results by calculating the Intersection over Union (IoU) ratio of all the detection results. The highest scoring detections are retained until the IoU value exceeds a set threshold. Therefore, the selection of the intersection and merger ratio threshold has an impact on the position of the localization candidate box. The purpose of filtering out overlapping boxes cannot be achieved if the threshold is too high; conversely, excessive features may be deleted if the threshold is too low, resulting in poor detection accuracy, which is calculated as in Eq (9):

$$\text{IoU}=\frac{A\cap B}{A\cup B}=\frac{A\cap B}{A+B-A\cap B}$$ (9)

Where *A* is the area of the candidate frame calibrated by the training set and *B* denotes the area of the face candidate frame. Eventually, the accuracy of the output candidate frame is judged based on the magnitude of the ratio.

The overall MTCNN loss function is represented by the weighted sum of three loss functions. The P-Net network for face recognition in the original MTCNN is trained using the cross-entropy loss function, and the input samples are computed as shown in Eq (10):

$$L^{\text{det}}=-(y_{i}^{\text{det}}\text{log}(p_{i})+(1+y_{i}^{\text{det}})(1-\text{log}(p_{i})))$$ (10)

Where $y_{i}^{\text{det}}$ the label set for the image and *P*_*i*_ denotes the probability of detecting as a face. The difference is calculated using the Euclidean distance, and the loss function of the target frame and the key point is shown in Eqs (11–12) [32]:

$$L^{box}=\left\|{\hat{y}}_{i}^{box}-y_{i}^{box}\right\|$$ (11)

$$L^{mark}=\left\|{\hat{y}}_{i}^{mark}-y_{i}^{mark}\right\|$$ (12)

${\hat{y}}_{i}^{box}$ denotes the bounding box coordinates after the algorithm output, $y_{i}^{box}$ is the real bounding box coordinates, ${\hat{y}}_{i}^{mark}$ is the key coordinate point within the algorithm output image, and $y_{i}^{mark}$ denotes the real coordinates of the key point. Eventually, as in Eq (13), the loss weights of each part are merged:

$$L=\text{min}\sum_{i=1\;}^{N}\sum_{j\in (\text{det},box,mark)}\alpha_{j}\beta_{i}^{j}L_{i}^{j}$$ (13)

where *N* is the total number of image training samples, $\alpha_{j}$ is the weight and $\beta_{i}^{j}$ is the sample type indicator. In this chapter set $\alpha_{det}=1$, $\alpha_{box}=0.5$, $\alpha_{mark}=0.5$ in P-Net,for O-net layer set $\alpha_{det}=1$, $\alpha_{box}=0.5$, $\alpha_{mark}=1$.

Since the traditional NMS algorithm directly removes the candidate boxes with IoU greater than the threshold, the process is highly potential to lose the information of the candidate boxes, which leads to insufficient learning of the model features due to data loss, and the detection effect fails to meet the expectation. To solve this problem, the chapter retains the candidate frames with IoU greater than the threshold, reduces their confidence level, and redefines the filtering rules, as shown in Eq (14) [33]:

$$s_{i}=\left\{\begin{array}{ll} s_{i}, & IoU(M,b_{i})\leq N_{t}\\ s_{i}(1-IoU(M,b_{i})), & IoU(M,b_{i})\geq N_{t} \end{array}\right.$$ (14)

where *N*_*t*_ is the threshold, *M* denotes the candidate frame with the highest confidence score, *b*_*i*_ denotes the face candidate frame, and *s*_*i*_ denotes the regression frame. The formula modifies the confidence of each candidate box that exceeds the threshold. After Algorithm 1 dynamically divides the computational resources of the edge server, ensuring that the minimum requirements of the face recognition algorithm of Algorithm 2 are fulfilled. As shown in Algorithm 2, if the updated new confidence is below the threshold, the candidate box is removed. The process iterates until all candidate boxes are labeled. Eventually, accurate face recognition results are output.

RETRACTED

**Algorithm 2:** Confidence Modified Face Recognition Algorithm

**Input:** face candidate frame set *b*_*i*_, regression frame set *s*_*i*_, candidate frame with the highest confidence score set *M*, threshold set *N*_*t*_

**Output:** Results of Face Recognition

 **Algorithm 1** Dynamically Segmenting Edge Servers (*S*)

 **For** *each i* **in** enumerate(*b*_*i*_) **do:**

  **IF** is_box_marked[i] **Then:**

   continue

  new_confidence = *M*[i] +*s*_*i*_[i] * delta_box_scores[i]

  **IF** new_confidence < *N*_*t*_ **Then:**

   is_box_deleted[i] = True

  *M*[i] = new_confidence

  is_box_modified[i] = True

  has_unmarked_box = True

 **End**

 **Return** Results of Face Recognition

Algorithm 2 is the confidence corrected face recognition algorithm, the time complexity of this algorithm can be divided into the following parts: iterate for each candidate box *b*_*i*_, the time complexity of this step is O(b), where *b* is the number of candidate boxes. Calculate the new confidence new_confidence. For each candidate box bi, the new confidence new_confidence needs to be calculated. This process includes the calculation of the confidence *M*[i], the regression box score *s*_*i*_[i] and other constants, assuming that the time complexity of calculating each new confidence is O(1). Determine whether to delete a candidate box, for each candidate box bi, it is necessary to determine whether the new confidence is lower than the threshold *N*_*t*_, and accordingly decide whether to delete the candidate box or not, this operation is completed in O(1) time. Update the candidate box set *M* and the labeling status, for each candidate box *b*_*i*_, if the confidence level needs to be modified, the candidate box set *M* and the labeling status are updated, and this operation is completed in O(1) time. To determine whether there are still unmarked candidate boxes in each iteration, it is necessary to check whether there are still unmarked candidate boxes to determine whether the iteration needs to continue, and this operation is completed in O(1) time. Therefore, the total time complexity of the algorithm is O(b).

RETRACTED

## 4. Experimental comparison and analysis

In this section, the algorithm comparison is done for edge service deployment, real-time face recognition task in IoT environment respectively and analyze the methodology proposed in this paper.

### 4.1 Experimental environment and data

The face detection experimental dataset used is the WiderFace face dataset, which is labeled with a total of 393,703 face instances containing a variety of face shooting angle images such as occlusion, aspect ratio imbalance, different stages of age, lighting changes, various other cases. The experimental dataset is divided into training and test sets with an overall ratio of 7:3, so the number of training sets is 7000, and the number of test and validation sets is 3000 each. In addition, the configuration of the simulation experiment hardware and software environment is shown in Table 3.

**Table 3:** Experimental environment.

Hardware Configuration	Parameters	Software Configuration	Parameters
CPU	Intel Core i7	Operating Systems	Windows10 64 位
GPU	GTX 2080Ti	Development Languages	Python 3.7
Hard Disk	1TB	Development Tools	Pycharm
RAM	32GB	Development Framework	TensorFlow 2.5

The model training parameters were configured to set the initial learning rate to 0.01, the weight decay coefficient to 0.0005, the batch size to 8, and the number of iterations to 200.

### 4.2 Evaluation indicators

For the experiments in this chapter, four commonly used classification metrics were chosen: *Accuracy* (*Acc*), *Precision* (*Pre*), and *Recall* (*Rec*), *F1*. As shown in Eq (15), *Acc* predicts the proportion of correctly classified samples to the total number of samples. *Pre* means the proportion of correctly predicted positive classes to the proportion of all predicted positive classes, as shown in Eq (16). As shown in Eq (17), *Rec* is the proportion of actual positive samples that are predicted to be positive to the proportion of actual positive samples that are predicted to be positive. The *F1* combines *Pre* and *Re*, as shown in Eq (18), where a higher *F1* score indicates that the proposed algorithm is more reliable.

$$Accuracy\;(Acc\text{)}=\frac{TP+TN}{TP+TN+FP+FN}$$ (15)

$$Precision\;(Pre\text{)}=\frac{TP}{TP+FP}$$ (16)

$$Recall\;(Rec)=\frac{TP}{TP+FN}$$ (17)

$$F1=\frac{2\times Pre\times Rec}{Pre+Rec}$$ (18)

where TP, TF, FP, and FN are denoted as confusion matrix values with specific meanings, as shown in Table 4.

RETRACTED

**Table 4:** Confusion matrix.

	Authenticity (positive)	Authenticity (negative)
Predicted value(positive)	TP	FN
Predicted value(negative)	FP	TN

In the confusion matrix, TP indicates True Positive, which means that the classifier correctly classifies positive example samples as positive examples. TF represents True Negative, in which the classifier correctly classifies negative samples as negative examples. FP denotes False Positive, where the classifier incorrectly classifies a negative sample as a positive example. FN stands for False Negative, meaning that the classifier incorrectly classifies a positive example sample as a negative example.

### 4.3 Performance evaluation of face recognition in TFREC

In TFREC two matrices, *W*, *V*, are used to map the inputs and outputs, the dimension of *W* is hidden*Input and the dimension of *V* is hidden*hidden. therefore, the space complexity of the simplified model is Eq (19), which reduces to Eq (20).

N=8(Hidden*Input+Hidden*Hidden+Hidden) (19)

$$Space\sim o(8(nm+n^{2}+n))$$ (20)

where n is the hidden size and m is the input size. The time complexity of the model is the number of operations on the number of model parameters, as shown by Eq (17):

$$Time\sim o(Epochs*8(nm+n^{2}+n))\sim o(n^{2})$$ (21)

where Epochs is the number of iterations, set to 200.

As shown in Table 5, TFREC is evaluated in terms of detection rate, response time. To highlight the performance of TFREC in this paper different IoUs are used to judge the face detection accuracy.

**Table 5:** Performance comparison of different IoU condition models.

IoU	Number of Successful Detection	Acc	Pre	Rec	F1	Total Time Consumption
0.50	2877	95.9%	97.4%	96.7%	97.0%	38.7S
0.55	2833	96.1%	98.3%	97.5%	97.9%	38.4S
**0.60**	**2949**	**98.3%**	**99.4%**	**98.5%**	**98.9%**	**27.3S**
0.65	2922	97.4%	98.5%	97.7%	98.1%	26.5S

As seen in Fig 5, the Pre rate of the TFREC algorithm gradually increases during the training process and stabilizes after 150 Epochs, finally reaching 99.4% and does not show substantial changes. Datasets used to provide Fig 5 were provided in S1 Table (see Supporting information).

**Fig 5:** Precision and Recall of TFREC algorithm.

According to the results in Table 3, when the IoU is 0.6, although the total elapsed time is not the least, it is significantly lower than the total elapsed time for IoU = 0.55 and close to the total elapsed time for IoU = 0.65. Remarkably, although the total elapsed time is not the least, the case with IoU of 0.6 performs the optimal in terms of accuracy. Thus, the comparison is so clear that the experiments that follow in this paper will only show the case when using an IoU of 0.6.

RETRACTED

Comparison experiments of TFREC algorithm with YOLOv3 [34], YOLOv5 [35], and AdaBoost [36], algorithm yielded a table of detection rates as shown in Table 6, and a graph of comparison of detection performance as shown in Fig 6.

**Fig 6:** Comparison of algorithm performance.

**Table 6:** Algorithm comparison experiments.

Algorithm	Number of Successful Detection	Acc	Pre	Rec	F1	Total Time Consumption
YOLOv3 [34]	2505	83.5%	91.3%	82.7%	86.7%	26.1s
YOLOv5 [35]	2580	86.0%	94.7%	85.5%	89.8%	26.7s
AdaBoost [36]	2652	88.4%	96.9%	83.1%	89.4%	25.8s
**TFREC**	**2949**	**98.3%**	**99.4%**	**98.5%**	**98.9%**	**27.3S**

To validate the correctness of the above analysis, the following hypothesis tests are done, based on the definition of H0 when there is no significant difference between the TFREC algorithm and the comparison algorithm, H1 when one algorithm outperforms the other and the difference is significant. The hypothesis experiments were carried out 100 times as shown in Table 7.

**Table 7:** Model hypothesis testing.

Comparison	TFREC Vs AdaBoost	TFREC Vs YOLOv5	TFREC Vs YOLOv3
Acc	H1 (Acc_TFREC_ >Acc_AdaBoost_)	H1 (Acc_TFREC_ >Acc_YOLOv5_)	H1 (Acc_TFREC_ >Acc_YOLOv3_)
Pre	H0 (Acc_TFREC_ = Acc_AdaBoost_)	H0 (Acc_TFREC_ = Acc_YOLOv5_)	H0 (Acc_TFREC_ = Acc_YOLOv3_)
Rec	H1 (Rec_TFREC_ >Rec_AdaBoost_)	H1 (Rec_TFREC_ >Rec_YOLOv5_ H0	H1 (Rec_TFREC_ >Rec_YOLOv3_)
F1	H1 (F1_TFREC_ >F1_AdaBoost_ H0)	H1 (F1_TFREC_ >F1_YOLOv5_ H0)	H1 (F1_TFREC_ >F1_YOLOv3_)

Based on the results of the experimental comparison, the comparison algorithm and the TFREC algorithm were compared in terms of face detection accuracy and overall detection time. Although the overall time for face detection using the TFREC algorithm is slightly higher than the comparison algorithm, the Pre rate reaches 98.3% and the Rec metric reaches 98.5%. Compared to the existing algorithms, both metrics were improved by about 10%, resulting in more successful detections. Also, the average face detection time is better than the rest of the algorithms. This means that there is a better balance between accuracy and detection time and the algorithm is able to detect faces faster and more accurately. Therefore, the conclusion to be drawn is that the model proposed in this paper shows promising results in face recognition and meets the needs of course teaching for dynamic face capture.

RETRACTED

### 4.4 Dynamic deployment performance evaluation in TFREC

Latency performance in edge computing is widely used as a quantitative metric in IoT environments that directly reflects the amount of time a system takes to process a task [37–39]. Efficient latency performance for IoT applications means faster response time and better real-time performance [40].

To further validate the low latency of TFREC, this paper performs a statistical analysis of evaluation metrics and compares it with other methods. Among them, Redundant Constrained Randomized Algorithm (RC) [41] improves the fault tolerance and reliability of the system by adding redundant computations. Average Randomized Algorithm (AR) [42] achieves load balancing by evenly distributing computational tasks and has low computational complexity. The Maximum Request Frequency (MRF) [43] algorithm, on the other hand, selects the most suitable edge nodes for processing based on the priority of the tasks to ensure timely completion of high-priority tasks, as shown in Fig 7.

**Fig 7:** Algorithmic delay comparison experiment.

For a certain amount of data and transmission rate, the deployment scenarios derived from different algorithms produce the same transmission delay. However, by analyzing the propagation delay, this paper finds that the TFREC algorithm reduces the delay to 72 milliseconds, which provides superior performance compared to other algorithms.

In IoT environments, the number of edge servers is typically limited and tends to be fixed. However, the number of users may increase as the demand increases. In this case, as shown in Fig 8, the TFREC algorithm exhibits a slow growth rate in terms of propagation delay compared to other algorithms.

**Fig 8:** Propagation delay versus number of students.

The TFREC algorithm is able to effectively reduce propagation delays and provide stable performance in edge computing environments by optimizing resource allocation and task scheduling. Although the number of students significantly exceeds the number of students actually teaching, the TFREC algorithm is still able to adapt and satisfy the large-scale task requirements and maintain favorable performance. Therefore, the teaching method reform model proposed in this paper is feasible.

## 5. Conclusion

This paper illustrates the wide application of IoT technologies in the field of education, especially the use of IoT devices and face capture services to improve teaching and learning in computer lab classes. In order to solve the problems of data processing and network latency, this paper proposes a teaching model of face recognition for IoT devices based on edge computing. The TFREC model uses a layer cascaded convolutional neural network for real-time recognition of the facial features of the students combined with edge computing to reduce the latency of the service, along with the use of a dynamic service deployment strategy to optimize the response time and resource utilization.

RETRACTED

## 6. Limitations and future work

The TFREC model achieves impressive accuracy in face recognition. However, misrecognition may persist in some cases of extreme conditions, as when a student is wearing a mask or an obscuring object such as a hat, where facial features may not be correctly recognised. To mitigate this challenge, the introduction of 3D face recognition algorithms will be explored in future research to improve overall error tolerance. In addition, future research should also focus on designing encryption algorithms for edge server transmission data to ensure secure data transfer during transmission and extending the TFREC model to additional teaching scenarios.

## Supporting information

S1 Dataset (XLSX)

S1 Table Datasets used to provide Fig 5. (XLSX)
